The article "HMGB1: a novel protein that induced platelets active and aggregation via Toll-like receptor-4, NF-κB and cGMP dependent mechanisms" was retracted in 2018. Reasons: errors in the methods; errors in the text; false authorship; unreliable results or conclusions.

# HMGB1: a novel protein that induced platelets active and aggregation via Toll-like receptor-4, NF-κB and cGMP dependent mechanisms

**DOI:** 10.1186/s13000-015-0348-3

**Published:** 2015-08-06

**Authors:** Xinyu Yang, Haichao Wang, Menmen Zhang, Jin Liu, Ben Lv, Fangping Chen

**Affiliations:** Depatment of Haematology, The Third Xiangya Hospital, Central South University, Changsha, Hunan PR China; Laboratory of Emergency Medicine, The Feinstein Institute for Medical Research, North Shore-LIJ Health System, Manhasset, NY 11030 USA; Department of Hemotology Xiangya Hospital, Central South University, Changsha, Hunan 410078 PR China

**Keywords:** HMGB1, Platelet aggregation, Thrombosis

## Abstract

**Background:**

Thrombotic diseases are a group of prevalent and life-threatening diseases. Selective inhibition of pathological thrombosis holds the key to treat variety of thrombotic diseases. The pathological thrombosis can be induced by either tissue necrosis and deregulated inflammation. HMGB1, as an important proinflammatory cytokine and a late mediator, also involves on thrombosis disease. However, the underlying mechanisms are not fully understood.

**Methods:**

Immunofluorescence, ELISA assay, Platelet Aggregation, Thromboelastogram (TEG) analyzes. Flow cytometric analysis and Western blot analysis were used to investigated the role of HMGB1 in platelet aggregation and obtained following observations.

**Results:**

By doing so, we obtained the following observations: i) Highly purified HMGB1 recombinant protein induces platelet aggregation and secretion in a dose-dependent manner in the presence of serum. ii) Low concentration of extracellular HMGB1 could synergistically promote subthreshold concentration of collagen or thrombin induced platelet aggregation. iii) Extracellular HMGB1 promoted platelet aggregation in a platelet-expressed GPIIb/IIIa-dependent manner. iv) We proposed that extracellular HMGB1 seems to promote the phosphorylation of GPIIb/IIIa and subsequent platelet aggregation via TLR4/NF-κB and cGMP pathway.

**Conclusions:**

In this study, we provide evidence for the hypothesis that HMGB1 interact with platelet might play an important role in the haemostasis and thrombotic diseases. Our research might be provide an interesting avenue for the treatment of thrombotic diseases in the future.

## Background

Evidence from basic and clinical medicine had clearly proven that there were complex interactions between inflammation and thrombosis. The pathogenesis of thrombosis remains complicated. Inflammation increases immune cells or endothelial cell release of procoagulant factors, such as cytokines, chemokines, adhesion molecules were released, tissue factor expression, platelet and endothelial activation [1], however, inflammation not only leads to activation of coagulation, and vice versa coagulation also considerably affects inflammatory activity and even augments inflammation, at present, the commonly accepted notion that inflammation and hemastasis are coupled by common activation pathway and feedback regulation system [2, 3], generally speaking, inflammation including sterile and infection- associated inflammation states, but the common features of the two in the process of inflammation are accompanied by cells necrotic and and immune cell activation [3].

The article "HMGB1: a novel protein that induced platelets active and aggregation via Toll-like receptor-4, NF-κB and cGMP dependent mechanisms" was retracted in 2018. Reasons: errors in the methods; errors in the text; false authorship; unreliable results or conclusions.

High mobility group box chromosomal protein 1 (HMGB1) was originally discovered as a chromatin-binding protein that could bend DNA. Such bending stabilizes nucleosome formation and regulates the expression of select genes upon recruitment by DNA binding proteins [4, 5]. Then, researchers discovered that extracellular HMGB1 can be released from necrotic cells, apoptotic cells or multiple immunocompetent cells and displayed a broad spectrum of biological activities [6, 7], importantly, extracellular HMGB1 play a critical role in activation of the innate immune response, by functioning as a chemokine facilitating movement of immune cells to sites of infection, as well as in functioning as a damage-associated molecular pattern (DAMP), activating other immune cells to secrete proinflammatory cytokines, thus promoting the immune response [8]. Recently, double-stranded RNA-dependent protein kinase (PKR) identified as a crucial regulator of inflammatory mediator HMGB1 released [9]. Present study clearly indicated that extracellular HMGB1 transmembrane signaling pathways main through Toll-like receptor (TLR)-4, TLR-2, and the receptor of advanced glycation end products (RAGE) [10, 11]. Moreover, HMGB1, as an important proinflammatory cytokine and a late mediator, also involves on thrombosis disease. A growing number of studies suggest that a potential role of HMGB1 in during thrombus development. In recent years, our study for the first time provided evidence that extracellular HMGB1, potentially through activation of transcription factors such as NF-κB, enhanced tissue factor (TF) expression and activities in vascular endothelial cells (ECs) and macrophages [12]. Moreover, another recent clinical study, doctors discoverd circulating HMGB1 has been shown to be independently associated with cardiac mortality in ST-segment elevation myocardial infarction [13].

Here, we found that either the resting platelets cytoplasm or the supernatant of activated platelets high expression of HMGB1 protein. Platelets play a central role in thrombosis, hemostasis, and inflammation. In addition to their known role in hemostasis and thrombosis, platelets also as immune cells, that forms a bridge between inflammation and thrombosis disease, play proinflammatory and procoagulant in vivo [14]. In addition, platelet also expression function TLR2, TLR4 and RAGE which implicated in the regulation of platelet adhesion, aggregation [15, 16]. For instance, recently reported that histone, which similar to HMGB1 protein as DAMP, could induce platelet aggregation and thrombin generation through platelet TLR2 and TLR4 [17]. Platelet activation and aggregation is essential for normal hemostasis and also plays a important role in thrombosis. In the past, although some researchers speculated that HMGB1 protein capable of activating platelets [18], but the mechanism was previously unclear. For the first time, we provided evidence that HMGB1 could direct induced platelets aggregation and secretion, moreover, extracellular HMGB1 could significantly promote other agonists-induced platelets aggregation. Furthermore, extracellular HMGB1 interact with platelets mainly depended on TLR4/NF-κB and cGMP-dependent pathway. Taken together, our experimental data suggest that HMGB1 protein this potent procoagulant function may contribute to pathogenesis of thrombosis.

The article "HMGB1: a novel protein that induced platelets active and aggregation via Toll-like receptor-4, NF-κB and cGMP dependent mechanisms" was retracted in 2018. Reasons: errors in the methods; errors in the text; false authorship; unreliable results or conclusions.

## Method

Recominant HMGB1 (rHMGB1) protein was expressed in Escherichia coli, and purified to homogeneity as described previously [19]. Purified HMGB1 was tested for endotoxin content by the chromogenic Limulus amebocyte lysate assay (Endochrome, Charles River, Wilmington, MA, USA), and contained < 500 pg endotoxin per microgram of rHMGB1. Blocking mAbs against human TLR2 (clone T2.5), TLR4 (HTA125), and isotype control (IgG2a, from eBioscience); mouse anti-human RAGE (R&D Systems, Catalog Number: MAB11451; 20 μg/ml), PE/FITC/Percp labeled anti-human IgG1, FITC-labeled anti-human PAC-1, PE-labeled anti-human CD62P, Percp-labeled anti-human CD61, FITC-anti-human labeled CD42b, PE-labeled anti-human CD41 (all from BD, USA), collagen (T-7009,100UN) and thrombin (Sigma), Ristocetin (Absin China), Rabbit polyclonal anti-HMGB1 antibodies (R&D Systems), human HMGB1 enzyme-linked immunosorbent assay (ELISA) kit was purchased from Shino-Test Corporation (Tokyo, Japan). Proteinase K (500 μg/ml Sigma-Aldrich). Sodium nitroprusside (SNP; 100 μM, Sigma, USA).

### Patients and samples

Blood samples were obtained from five healthy donors and the patient with Glanzmann thrombasthenia (GT) is a 40-year-old woman, the detailed data about laboratory molecular biological diagnostic had published in Blood [20], the institutional ethics committee of the third Xiangya hospital of central south university approved this study, all patients and healthy donors gave their informed consent in accordance with the declaration of Helsinki. Blood sampling, PRP preparation and platelet isolation, all peripheral venous blood was collected from patients or healthy human volunteers by puncture with a 19-gauge needle, Storage tube contain 3.8 % trisodium citrate (9:1 blood-to-citrate ratio, BD Vacutainer™ tubes). PRP preparation and platelet isolation processed as described previously [17]. PRP was centrifuged at 1000 rpm for 10 min at at room temperature (RT) in the presence of 1 μg ml^-1^ PGE_1_ (Sigma-Aldrich) and next 3000 rpm for 10 min then washed in washing buffer (140 mM NaCl, 10 mM NaHCO_3_, 2.5 mM KCl, 0.5 Mm Na_2_ HPO_4_, 1 mM MgCl_2_, 22 mM sodium citrate, 0.55 mM glucose, 0.35 % BSA, pH6.5). Finally, washed human platelets (WPs) were resuspended in Tyrode’s buffer (Tyrode buffer composition was 10 mmol/L of HEPES pH7.5, 140 mmol/L of NaCl, 2.7 mmol/L of KCl, 0.2 mmol/L of Na_2_HPO_4_, 12 mmol/L of NaHCO_3_, 5.5 mmol/L of D-glucose, and 1 mmol/L of MgCl_2_).

The article "HMGB1: a novel protein that induced platelets active and aggregation via Toll-like receptor-4, NF-κB and cGMP dependent mechanisms" was retracted in 2018. Reasons: errors in the methods; errors in the text; false authorship; unreliable results or conclusions.

### Immunofluorescence

WPs were resuspended in Tyrode’s buffer, then platelets of two groups were fixed with 1 % paraformaldehyde and cytospined after by adding thrombin, the processed platelets incubated overnight with rabbit polyclonal anti-HMGB1 antibodies and Rabbit polyclonal anti-actin antibodies. The washed platelets were incubated for 1.5 h at RT with the secondary Ab Alexa Fluor 488 or 568 (Molecular Probes) at a dilution of 1:500 followed by 3 washes in PBS. Images of platelets were visualized by fluorescent microscopy (Nikon), shutter and image acquisition were controlled by MetaMorph software (MDS Analytical Technologies).

### ELISA assay

The addition or not addition of thrombin (0.2 U/ml) to WPs, respectively measured protein of HMGB1 in the supernatant and pellet after platelet activation, the rest platelet as control. HMGB1 plasma concentrations were measured using the HMGB1 ELISA Kit II according to the manufacturer’s protocols. The lower limit of quantification for the assay was 0.2 ng/mL for HMGB1. Each sample was run in duplicate and the mean concentration was determined.

### Platelet aggregation

Aggregation of platelets were finished in 30–40 min when fresh blood from healthy volunter was collected, the method was optically monitored in a Data 4-chamber aggregometer (Chrono-Log Lumi-aggregomete) at 37 °C, magnetic stick at a constant stirring rate of 1200 rpm, PRP was centrifuged at 1000 rpm for 10 min at at RT, adjust the number of platelets (200–250 × 10^9^/mL) in WPs, Light ray transience through WPs is 100 %, but through Tyrode’s buffer it is 0 % due to differing optical density. WPs (200 μl) was poured into glass tubes in the presence of a magnetic stick, platelet aggregation was determined by adding 50 μl of HMGB1 or other agonists, including Thrombin (0.2 unit/ml), Collagen 0.3 μg/ml, Ristocetin (RIS 1.25 mg/ml), Albumin (μg/ml) was set as negative control.

The article "HMGB1: a novel protein that induced platelets active and aggregation via Toll-like receptor-4, NF-κB and cGMP dependent mechanisms" was retracted in 2018. Reasons: errors in the methods; errors in the text; false authorship; unreliable results or conclusions.

### Thromboelastogram (TEG) analyzes

A whole blood kaolin-activated thromboelastogram (TEG) analyses was run in a CFMSTM thromboelastography(China), TEG experiment with CFMSTM thromboelastograp General Cup Test Kit (viscosity measuring). The basic TEG parameters include reaction time R, angle of alpha (α) and Maximum Amplitude (MA). With whole blood 2 ml from health donors storaged in tube contained 3.8 % trisodium citrate (9:1 blood-to-citrate ratio, BD Vacutainer™ tubes). take 1 ml of whole blood to the first reagent reacting vessel (contain kaolin clay) of the kit, a final concentration of 1 μg/ml HMGB1 protein were added or not added to some vessels, very slowly with sufficient mixing, waiting for 5 min, then, adding 20 μl CaCl_2_ (the second reagent reacting vessel) to the bottom of reaction cups, At the time the reaction was started, 320 μL of citrated whole blood was added to the cup, and the recording was initiated. All TEG analyzes were performed within one hour after sample collection.

### Flow cytometric analysis

Platelets in Tyrode buffer were incubated with HMGB1 for 10 min at 37 °C and then in the presence of 2.5 mmol/L of CaCl_2_. Albumin (60 μg/ml) as control, next, For P-selectin and PAC-1 evaluation, platelets were diluted in HBS and fixed with adding paraformaldehyde (final concentration of 1 %) in at 37 °C for 5 min; afterward, they were washed and incubated in HBS with 1 % BSA containing FITC-labeled PAC-1 or PE-labeled CD62P or Percp-labeled CD61 for 30 min, in some experiments, platelets were pre-incubated with anti-TLR2 mAbs, anti-TLR4 mAbs, anti-human RAGE mAbs or IgG2a (50 μg/mL) for 20 min at RT; then washed again and resuspended in HBS with 1 % BSA, For analysis patients with GT, platelets were washed and incubated in HBS with 1 % BSA containing Percp-labeled CD61 or FITC-labeled CD42b or PE-labeled CD41a, PE/FITC/Percp labeled anti-human IgG1 as isotype control antibody, expression was analyzed using a FACSCalibur flow cytometer (BD Biosciences).

### Measurement of platelet cGMP, cAMP levels

WPs pre-incubated with or without blocking mAbs anti-TLR2, anti-TLR4, anti-human RAGE or IgG2a mAbs (60 μg/mL) for 10 min at 37 °C respectively. HMGB1 was added to WPs that were stirred at 37 °C in a platelet aggregometer for 5 min. and the reaction stopped by addition of ice-cold 12 % (w/v) trichloroacetic acid. Samples were mixed and centrifuged at 2000 g for 15 min at 4 °C and the supernatant was extracted four times with water-saturated diethyl ether. The samples were lyophilized (≤-20 °C) and concentration determined using a cGMP, cAMP enzyme immunoassay kit from Amersham Biosciences. Results are expressed as mean ± SD.

The article "HMGB1: a novel protein that induced platelets active and aggregation via Toll-like receptor-4, NF-κB and cGMP dependent mechanisms" was retracted in 2018. Reasons: errors in the methods; errors in the text; false authorship; unreliable results or conclusions.

### Western blot analysis

WPs lysates (10^9^ cells/mL) were prepared in loading buffer (62.5 mM Tris–HCl at pH 6.8, 25 % glycerol, 2 % SDS, 0.01 % bromophenol blue and 5 % 2-mercaptoethanol) in the presence of a protease inhibitor cocktail containing 1 mM AEBSF, 2 μg/ml aprotinin, 1 μg/ml leupeptin. Equal volume of platelet proteins were resolved by 12 % sodium dodecyl sulfate-polyacrylamide gel electrophoresis (SDS-PAGE). The proteins were transferred to a PVDF membrane (Millipore) by semidry transfer, Antibodies to human HMGB1mAb (R&D Systems), and Actin(Cell Signaling). Mouse anti-IκBα, rabbit anti-phospho IκBα were from Abcam (UK).

### Statistical evaluation

All data are presented as mean ± standard deviation (SD). Statistical analysis was performed by the Student *t*-test or ANOVA as appropriate. *P* < 0.05 was considered to be statistically significant.

## Result

### Resting human platelets express cytoplasmic HMGB1, activated platelet release of HMGB1

In our study, we discovered that HMGB1 protein was high expressed in washed human platelets (WPs). Next, we further confirmed HMGB1 protein were mainly located in the intracellular when it in the resting state by immunoblotting or ELISA test, rarely HMGB1 protein exist in the plasm, the resting platelets in pellets contain HMGB1 protein were 10.27 ± 1.01 ng/10^9^ platelets, the extracellular fluid of platelets contain HMGB1 protein were only 0.19 ± 0.13 ng/10^9^ platelets, however, when added simultaneously with the platelet agonists thrombin (0.2 U/ml), thrombin-stimulated platelets contain HMGB1 protein in pellets were changed to 2.39 ± 0.70 ng/10^9^ platelets and extracellular HMGB1 protein levels in the supernatant significantly increase to 7.86 ± 1.10 ng/10^9^ platelets. Compared to resting platelets, the level of HMGB1 protein both in pellets and in supernatant had statistically significant difference after thrombin-stimulated platelet (Fig. 1). The results are consistent with other researcher previous finding [18]. The purpose of releasing of the HMGB1 protein during platelet activation is still not clear, what kind of role it will play in platelet activation is our next step focal point.

**Fig. 1:** Platelets express HMGB1. **a** Representative immunoblot of HMGB1 expressions in WPs (1 × 10^9^/ml) from five different health donors, Western blot analysis of extracts HMGB1 protein by HMGB1 polyclonal antibodies. **b** HMGB1 was assessed by ELISA in pellets and supernatant of WPs that either resting or adding thrombin (0.2 U/ml). After WPs were activated, the concentration of HMGB1 in pellets or in the supernatant signicantly different from the resting WPs group (*n* = 5, *P < 0.01). **c** WPs incubated with or without (negative controls) rabbit polyclonal-anti-HMGB1 (blue) in combination with rabbit-anti-Actin (red), respectively. Images under fluorescent microscopy, the results indicated that the resting WPs high expression of HMGB1 protein

High conceration of rHMGB1 protein directly induce platelet aggregation and low dose of rHMGB1 protein potentiates other agnoists-induced platelet aggregation activated platelets release of HMGB1 protein, which is whether similar to thromboxane A2 (TXA2), ADP, or Polyphosphates (Polyp) that were released from activation of platelets then involved in increasing platelet-self activation or enhances blood clotting reactions.so we first examined the effect of rHMGB1 protein on platelet aggregation, test results were amazing and revealed that stimulation of WPs with various levels of HMGB1 protein (0 to 160 μg/ml) led to a concentration dependent induction of platelet aggregation (Fig. 2a, b). A few micrograms of (1–5 μg/ml) rHMGB1 protein alone can not induce platelet aggregation, while as the protein concentration increasing, compared to control group (ALB), rHMGB1 protein (10 μg/ml) induce platelet aggregation rate were 10.3 % ± 4.7 % (*n* = 5, *P* < 0.05), because LPS stimulation also can induce platelet secretion and promote aggregation. we wish to exclude the possibility that contaminating LPS in the HMGB1 preparation (<500 pg LPS per microgram of HMGB1) contributes to the observed increase platelet aggregation. Accordingly, an effective inhibitor of LPS, polymyxin B (PMB), was employed in parallel experiments. when given at a low concentration (500 pg/ml), LPS not direct induce platelet aggregation, LPS effect completely abrogated after rHMGB1 by co-incubation with PMB (1 μg/ml). We found that rHMGB1 (40 μg/ml)-induced platelet aggregation was not decreased by PMB (Fig. 2c, d). in contrast, rHMGB1-induced platelet aggregation generation was severely impaired in the presence of the proteinase K (PK) which dissolves the rHMGB1 proteins and destroy the native protein structure. When HMGB1 pre-incubated with PK (500 μg/ml) then the platelet aggregation drop markedly from 47.4 % ± 5.2 % to 11.7 % ± 5.7 % (*n* = 5, *P* < 0.05). We acquired the same result that treatment HMGB1 via rreversible thermal denaturation that changed the protein high-grade structure with high temperature cannot induce platelet aggregation.

The article "HMGB1: a novel protein that induced platelets active and aggregation via Toll-like receptor-4, NF-κB and cGMP dependent mechanisms" was retracted in 2018. Reasons: errors in the methods; errors in the text; false authorship; unreliable results or conclusions.

**Fig. 2:** HMGB1 directly induces platelet aggregation, results are expressed as mean ± SE. The data shown here are representatives of at least five experiments from different donor. **a** Various concentrations of HMGB1 protein induced platelet aggregation curves, albumin (ALB) is negative control, (**b**). Record data are means the maximum platelet aggregation rate induced by HMGB1 (*n* = 5, *P < 0.05 vs. ALB group). **c** and **d** The effects of PMB or proteinase K on HMGB1-induced platelet aggregation curves. HMGB1 (40 μg/ml) were pretreatmented with PMB (1 μg/ml) or proteinase K (500 μg/ml PK) for 10 min at RT, or thermal denaturation of HMGB1 (TD) at 100 °C for 10 min respectively, rHMGB1-induced platelet aggregation were obvious inhibited by PK or treatment of thermal denaturation, but not affected by PMB. (*n* = 5, *P > 0.05; **P < 0.05. vs HMGB1 group)

Hatada et al. from Japan reported that disseminated intravascular coagulation (DIC) was associated with significantly high plasma HMGB1 and the highest plasma levels of HMGB1 can be achieved 16.58 ± 11.01 ng/ml in non-survivors patients with organ failure [21]. Accordingly this reports, we speculated that the highest plasma levels of HMGB1 protein in local inflammation, necrotic tissue or worn-out organs may achieve a few micrograms. now that low dose of HMGB1 protein (1 μg/ml) which alone incapable of inducing platelet aggregation, it was unknown that low level of HMGB1 protein together with other agonists whether had best cooperation effects. Therefore, when adding simultaneously with subthreshold concentrations of agonists thrombin (0.2 U/ml) or collagen (0.3 μg/ml), we discovered that HMGB1 increased the maximum platelet aggregation rate induced by subthreshold level of thrombin or collagen (Fig. 3a, b). These results were further confirmed by thromboelastogram (TEG) analyzes. when the whole blood were pretreatmented with HMGB1, the Maximum Amplitude (MA) in TEG, which represents fibrin and platelet aggregation, was significantly enhanced from 61.7 ± 6.8 mm to 75.6 ± 7.5 mm (*n* = 5, *P* < 0.05) (Fig. 3c, d). Meanwhile, from the the result of TEG, we found that the cloting reacting time (R min), which represents the rate of initial fibrin formation and is related to plasma clotting factors and circulating inhibitory activity, gotten slightly extended but between of two have no statistical differences (data not show). These result suggested that HMGB1 incapable of initiating coagulation through directly activate coagulation factor.

**Fig. 3:** HMGB1 enhanced agonists-induced platelet aggregation. **a** A subthreshold concentration of thrombin (0.2 U/ml) or collagen (0.3 μg/ml) was added to WPs which were preincubeted with HMGB1 (1 μg/ml) or ALB for 10 min at 37 °C, above is representive platelet aggregation curve. **b** Data are expressed as mean ± SE, HMGB1 (1 μg/ml) that significantly enhancing thrombin or collagen-induced platelet aggregation rate (*n* = 5, *P < 0.05. vs collagen + ALB or thrombin + ALB group respectively). **c** Representative map of thromboelastogram (TEG) analyzes, the whole blood prior stimulated with HMGB1 (1 μg/ml) for 10 min at 37 °C, this one Maximum Amplitude (MA) was 77.1 mm. **d** Analyzing quantitative data from C, the MA of the HMGB1 group were enhanced (*n* = 5, *P < 0.05. vs HMGB1 + ALB)

The article "HMGB1: a novel protein that induced platelets active and aggregation via Toll-like receptor-4, NF-κB and cGMP dependent mechanisms" was retracted in 2018. Reasons: errors in the methods; errors in the text; false authorship; unreliable results or conclusions.

### Measurement of ATP release and expression of P-selectin

Platelet secretion is critical in amplifying platelet activation and in stabilizing thrombus. It is well established that activation platelets secreted ATP from dense granules. In addition, P-selectin which is a member of selectin family of cell surface receptor and also known as platelet activation dependent granule external membrane protein. To determine HMGB1simulated platelet secretion, we first measured the release of ATP in the supernatant in HMGB1 stimulated WPs (Fig. 4a). The results indicated that a few micrograms of HMGB1 alone was suficient to induce platelets release of ATP, when WPs incubated with HMGB1 protein (1 μg/ml), measured ATP in the supernatant were 0.70 ± 0.08 nmol/mL, while the control (add Buffer) were only 0.53 ± 0.07 nmol/ml, ATP secretion was sinificantly enhanced in HMGB1-stimulated WPs. Similarly, in order to exclude the possibility that contaminating LPS contributes to the observed increase platelet secretion. LPS (500 pg) was able to slightly increase ATP in WPs (P > 0.05), co-incubation with PMB (1 μg/ml) completely blocked LPS-mediated platelet secretion, but did not change rHMGB1-induced platelet secretion (Fig. 4d).

**Fig. 4:** **a** ATP release was determined (by ATP Assay Kit) in rHMGB1-incubated WPs (1 × 10^9^/ml), WPs were treated with rHMGB1 (1-80 μg/ml) in an aggregometer (1200 rpm) for 5 min at 37 °C (*n* = 6, *P < 0.05 vs. rest group). **b** WPs were pre-incubated with various concentrations of HMGB1 protein for 10 min, fixed with paraformaldehyde, then incubated with HMGB1 in the presence of a monoclonal anti-human P-selectin Ab or control mouse IgG (Rest) for 30 min at room temperature. (*n* = 6, *P > 0.05; **P < 0.05, vs. rest group). **c** Flow cytometric determination of P-selectin expression level. **d** The effects of LPS and PMB on rHMGB1-induced ATP in WPs. (*n* = 6, *P > 0.05; **P < 0.05, vs. rest group)

During platelet activation, P-selectin is translocated from intracellular granules (α-granules) to the external membrane, it expression on platelets determines size and stability of platelet aggregates [22]. HMGB1 inducing platelets P-selectin expression and the results suggested that HMGB1 also stimulated platelets α granule secretion (Fig. 4b, c). measured P-selectin expression level in HMGB1-incubated (1 μg/ml) WPs were 14.0 % ± 5.3 %, although P-selectin expression level had a slightly increase while the results between the two (control group, 6.4 % ± 4.8 %) had no statistical difference, higher dose of HMGB1 (10 μg/ml) produced a significant increase P-selectin-positive platelets. in a words, these results revealed that HMGB1 stimulate platelet both dense and α granule.secretion.

The article "HMGB1: a novel protein that induced platelets active and aggregation via Toll-like receptor-4, NF-κB and cGMP dependent mechanisms" was retracted in 2018. Reasons: errors in the methods; errors in the text; false authorship; unreliable results or conclusions.

### HMGB1-induced platelet aggregation depends on GPIIb-IIIa complex activation

The linking of the platelets via fibrinogen brings about platelet aggregation. The glycoprotein (GP) layer of the platelet, such as GPIb, GPIIb-IIIa or GPIa-IIa and so on, plays a very important role in platelet function including adhesion and aggregation [23]. Normal primary platelet aggregation mainly requires agonist-mediated activation of membrane GPIIb-IIIa, which directly interact with fibrinogen mediated platelet-platelet interactions, may be involving other GP. We unknown whether HMGB1-induced platelet aggregation also mediated via GPIIb-IIIa which triggered an outside-in signaling cascade. Next, we found a patients with Glanzmann thrombasthenia (GT), who was first diagnosed and molecular biological analyses showed a severe reduction in surface GPIIb-IIIa receptors in platelets [20]. (Figure 5a) (the details of diagnosis information we published in Blood, 1996). The most common of GT patients, was characterized by a defective platelet aggregation in response to agonists that depended GPIIb-IIIa receptors. results from we found that HMGB1 was incapable of inducing platelet aggregation in patients with GT, as positive control, ristocetin can stimulate GT patients platelet aggregation via characterizing the interaction of von Willebrand factor (VWF) with platelets GPIb [24]. Furthermore, to obtain more direct evidence for such a linkage that the activated conformation of GPIIb-IIIa formation on HMGB1-mediated platelets. We confirmed PAC-1 expression on HMGB1-stimutited platelets by flow cytometry. The results indicated that a significant increase of PAC-1 expression on HMGB1-stimulated platelets. All these results indicated that signaling in HMGB1-induced platelet aggregation also depending an increased affinity of integrin GP IIb/IIIa.

**Fig. 5:** HMGB1-induced platelet aggregation depends on GPIIb-IIIa. **a** the results of the flow cytometric analysis of a patients with Glanzmann thrombasthenia (GT), CD41a and CD61 only expressed 0.7 % and 0.5 % respectively. **b** HMGB1 was incapable of promoting platelet aggregation in patients with GT, as positive control, Ristocetin (1.25 mg/ml) can promote platelet aggregation. **c** Representative graph of Flow cytometry analysis of PAC-1. **d** HMGB1 up-regulated the expression of platelet surface Pac-1 (*n* = 5, *P < 0.01 vs. ALB)

The article "HMGB1: a novel protein that induced platelets active and aggregation via Toll-like receptor-4, NF-κB and cGMP dependent mechanisms" was retracted in 2018. Reasons: errors in the methods; errors in the text; false authorship; unreliable results or conclusions.

### HMGB1 induced platelet activation depended TLR4

At present, it is very clear that HMGB1 transmembrane signaling pathways mainly depend TLR-4, TLR-2, and RAGE [10, 11]. To evaluate the potential roles of these receptors in HMGB1-induced platelet activation, the involvement of TLR2, TLR4 and RAGE in HMGB1-induced platelets aggregation or secretion was investigated by specific neutralising antibodies. WPs were preincubated with various concentration of blocking Abs directed against these receptor for 20 min respectively and then rHMGB1 (40 μg/ml) was added to platelet aggregation test. Our results suggested that HMGB1- induced platelet aggregation was obviously decreased after in the presence of increasing concentrations of anti-TLR4 Abs. in contrast, the irrelevant control antibody (IgG2a) or anti-TLR2 Abs and anti-RAGE Abs did not alter HMGB1-induced platelet aggregation even when given the same concentrations. Similarily, change in expression of P-selectin was consistent with above observations. WPs pretreatmented with anti-TLR4 (50 μg/mL) for 20 min and then HMGB1 (40 μg/mL) was added to measure P-selectin expression, the exposure of P-selectin were reduced from 52.8 % ± 5.6 % to 24.7 % ± 6.1 % in HMGB1-simulated WPs (*P < 0.05) (Fig. 6f, g), meanwhile, we examined the effect of the simultaneous with all neutralizing antibodies and the results indicated incapable of any further enhance the inhibition effect (data not shown). In conclution, above results suggested that the stimulatory effect of HMGB1 on platelet activation is, at least in part, TLR4 dependent.

**Fig. 6:** HMGB-induced platelet activation dependent on TLR4, the data shown here are representatives of at five experiments from different donors. Results are Means ± SD. Prior to stimulation with HMGB1 (40 μg/ml), WPs were pretreatmented with various conceration of anti-TLR4 Abs, anti-TLR2 Abs, anti-RAGE Abs, or irrelevant control concerationg IgG2a in an aggregometer (1200 rpm) for 20 min respectively. Representative aggregation curves with anti-TLR4 (**a**), anti-TLR2 (**b**), anti-RAGE (**c**) or IgG2a (**d**) are shown. **e**, **f** Statistical analysis of the maximum platelet aggregation rata (*n* = 5, *P < 0.05, **P < 0.01, vs IgG2a) and P-selectin expression data (*n* = 5, *P < 0.05 vs IgG2a). **g** Representative flow cytometric data showed that reduced HMGB1-induced P-selectin expression

The article "HMGB1: a novel protein that induced platelets active and aggregation via Toll-like receptor-4, NF-κB and cGMP dependent mechanisms" was retracted in 2018. Reasons: errors in the methods; errors in the text; false authorship; unreliable results or conclusions.

### HMGB1 stimulates platelet aggregation by blocking the activity of nitric oxide/cGMP signaling

cAMP and cGMP were an important secondary messenger in platelet, cAMP-dependent protein kinase A and cGMP-dependent protein kinase substrates translate prostacyclin and nitric oxide signals into a block of platelet adhesion, granule release, and aggregation [25] to investigated intracellular cAMP and cGMP levels in HMGB1-stimulated WPs by immunoassay kit, we measured cAMP and cGMP level in HMGB1-stimulated WPs and interesting found cGMP levels decreased in a dose-dependent manner after presence of serum, however, the changed of cAMP levels had no statistical difference (Fig. 7a). The reduced of cGMP levels play what a role in HMGB1-stimulated platelet was unknow, so next, we prior adding cGMP analogs 8-pCPT-cGMP or cGMP-elevating NO donor SNP WPs (sodium nitroprusside) to WPs respectively. The result indicated that HMGB1 (40 μg/ml)- induced the maximum platelet aggregation rate was significantly reduced after platelets incubation with 8-pCPT-cGMP, or SNP (ALB used as a negative control) (Fig. 7b, c). Above results suggested that nitric oxide/cGMP signaling play a suppressing role in HMGB1-stimulated platelets activation. On the other hand, we previous studies indicated that HMGB1 signals by binding to TLR4 to induce platelets activation, to investigate whether TLR4, TLR2 and RAGE receptors may be upstream of the cGMP signaling pathway. We examined the effect of anti-TLR4 Abs, anti-TLR2 Abs and anti-RAGE Abs on HMGB1-induced cGMP production respectively, our studies revealed that HMGB1-induced cGMP level change was almost completely abolished by anti-TLR4 Abs, there were also slightly inhibited by anti-TLR2 and anti-RAGE, but both of them have no statistical differences (Fig. 7d). Together with previous found showed that HMGB1 induced human platelets activation main depending on TLR4 /cGMP axis and the results futher supported our previous discover.

**Fig. 7:** cGMP levels decreased in HMGB1-induced WPs (**a**) WPs (10^8^/ml) under high shear (1200 rpm) in an aggregometer and stimulated with HMGB1, 37 °C 10 min, cGMP and cAMP concentrations were determined by using a immunoassay kit (*P < 0.01, **P > 0.05 vs control). **b**, **c** WPs were pretreatmented with 8-pCPT-cGMP (200 μM), or SNP (100 μM) in an aggregometer (1200 rpm) at 37 °C for 10 min and then addition of HMGB1 (40 μg/mL), platelet aggregation generation was then evaluated (*n* = 5, *P < 0.05 vs ALB). **d** WPs were preincubated with mouse IgG2a or anti-TLR4, anti-TLR2 mAbs or anti-RAGE mAbs (50 μg/ml) at 37 °C for 10 min and then incubated with HMGB1 (40 μg/mL) for 10 min. cGMP level was evaluated (*n* = 5, *P < 0.05 vs IgG2a). Results are the Means ± SD of at least 5 experiments

The article "HMGB1: a novel protein that induced platelets active and aggregation via Toll-like receptor-4, NF-κB and cGMP dependent mechanisms" was retracted in 2018. Reasons: errors in the methods; errors in the text; false authorship; unreliable results or conclusions.

### NF-κB inhibitors impair HMGB1-induced platelet activation responses

NF-**κ**B is a major transcriptional regulator of genes involved in survival, proliferation and inflammation of cell. HMGB1 itself may signal through TLR4 and TLR2, and via RAGE activation of these receptors results in the activation of NF-**κ**B, which involved in regulation of inflammation and activation of immune cells [11], to evaluated the role of NF-κB in HMGB1-induced platelet activation. WPs preincubated with various conceration of NF-κB inhibitors BAY 11-7082 before presented of HMGB1. the results suggested that HMGB1 mediated maxim aggregation rate in WPs was markedly inhibited by BAY 11-7082 in a dose-dependent manner (Fig. 8a). It was meaning that NF-κB activation playing a stimulatory role in HMGB1-induced platelets activation. Furthermore, Fig. 8b shows that HMGB1- induced WPs activation resulted in IκBα phosphorylation and more than a 70 % degradation of IκBα (Fig. 2b). both events were prevented by platelets preincubation the with BAY 11-7082, a specific inhibitor of NF-κB activation that prevents IκBα phosphorylation [26] meanwhile, it was interesting discovered that the cGMP level significantly elevate in WPs that pre-treatmented with increasing conceration of BAY11-7082 before adding HMGB1. (Fig. 8c, d) in order to support above results, we estimated the levels of PAC-1 expression by flow cytometry, HMGB1-mediated PAC-1 expression were significantly decreased in BAY 11-7082-treated platelets (data not show), In addition, we futher confirmed the TLR4/NF-κB signal passway and show that anti-TLR4 similar to BAY 11-7082 also showed a similar inhibitory activity against IκBα phosphorylation.however, guanylate cyclase (sGC) inhibitor ODQ can increase IκBα phosphorylation that impaired by BAY 11-7082 in HMGB1 stimulated platelets (Fig. 8f). Together, these observations suggest that TLR4/ NF-κB axis is involved in the regulation of “inside out” signal depending cGMP signal during in HMGB1-stimulated platelet activation.

**Fig. 8:** NF-κB inhibitors impair HMGB1-induced platelet activation responses and elevated cGMP level. **a**, **b** NF-κB inhibitors impair platelet aggregation induced by HMGB1, WPs were treated with the indicated concentrations of BAY11-7082 in an aggregometer (1200 rpm) at 37 °C for 5 min and then stimulated with HMGB1 (*n* = 5, *P < 0.01 vs ALB). **c** HMGB1 induce IκBα phosphorylation and degradation, WPs were treated with various dose of HMGB1 for 5 min 37 °C, then Lysates were immunoblotted with an anti- IκBα Ab. **d** WPs preincubation with BAY 11-7082 under high shear (1200 rpm) in an aggregometer for 5 min and then stimulated with HMGB1 (40 μg/ml) for 5 min, HMGB1 induce IκBα phosphorylation can be blocked by BAY 11-7082. (*n* = 4, *P* < 0.01 vs control). **e** Effects BAY 11-7082 on HMGB1-induced cAMP and cGMP, WPs pretreatment with BAY11-7082 in an aggregometer and stimulated with HMGB1 (40 μg/ml) for 5 min before termination of the reaction and then cAMP and cGMP enzyme immunoassays were performed. BAY11-7082 significantly increased cGMP accumulation in a dose dependent manner. (*n* = 4, *P < 0.01 vs. control). **f** Effects of a-TLR4, SNP, BAY 11-7082 or ODQ on HMGB1-induced IκBα phosphorylation. WPs were stirred in an aggregometer with above materials for 5 min prior to the addition of HMGB1 (40 μg/ml). a-TLR4 (50 μg/ml), SNP (100 μM) ODQ (20 μM) and BAY 11-7082 (40 μM), measured IκBα phosphorylation level, all immunoblots are representative of 3 to 4 similar experiments

The article "HMGB1: a novel protein that induced platelets active and aggregation via Toll-like receptor-4, NF-κB and cGMP dependent mechanisms" was retracted in 2018. Reasons: errors in the methods; errors in the text; false authorship; unreliable results or conclusions.

## Discussion

Emerging evidence has suggested a potential role for extracellular role of HMGB1, which was identified as a proinflammatory cytokine and a late mediator of sepsis. Beijnum et al first discovered that extracellular HMGB1 levels were elevated in human atherosclerotic plaques, but not in normal arteries [26]. Then, many studies demonstrated massive accumulation of HMGB1 in the systemic circulation would promote the development of DIC [21, 27] next, our research group first confirmed that HMGB1 elevated human vascular endothelial cell tissue factor expression and may be involved in the pathophysiology of atherothrombosis [12]. Recently another a clinical validation studies showed that a pathogenic relationship between extracellular HMGB1 and thrombosis has been proposed that circulating concentration of HMGB1 on admission may be a potential and independent predictor of cardiovascular mortality [13].

Here, our study shows for the first time that HMGB1 induced human platelets aggregation and secretion in a concentration-dependent manner. Furthermore, HMGB1 stimulates platelet secretion or aggregation mainly, at least in part, via the TLR4 dependent mechanisms. As mentioned above, extracellular HMGB1 is known to interact with three cell surface receptors: TLR4, TLR2, and RAGE. Known endogenous ligands released from damaged tissues such as heat-shock proteins [28], histone [17], and extracellular matrix fragments [29] all interact with TLR2 or TLR4, there is also considerable emerging evidence demonstrating that TLR4, may play a critical role in inflammation and autoimmunity, are predominantly involved HMGB1-mediated activation of innate immune cells [10]. For instance, TLR4 involved in regulation of HMGB1-induced neutrophil extracellular trap formation [30] or HMGB1-mediated platelet-tumour cell interaction [31]. Meanwhile, platelet expression of Toll-like receptor that was regarded as the link between “danger” ligands and inflammation [32]. Particularly, platelets depended express functional TLR4, which is MyD88-dependent or MyD88- independent pathways, plays a major role in platelet adhesion and promoting pro-inflammatory cytokine production [33]. Our experimental data suggested that HMGB1 interact with platelets via TLR4 and then triggered inside-out signaling in platelets, the conclusion are supported by our data that when anti-TLR4 mAbs, anti-TLR2 mAbs and anti-RAGE mAbs are all presenting in platelets only the HMGB1-stimulated effect is suppressed by anti-TLR4.

The article "HMGB1: a novel protein that induced platelets active and aggregation via Toll-like receptor-4, NF-κB and cGMP dependent mechanisms" was retracted in 2018. Reasons: errors in the methods; errors in the text; false authorship; unreliable results or conclusions.

In addition, our data suggested HMGB1 signaling were transmitted from TLR4 to GPIIb/IIIa and then triggers close cell-to-cell contact between platelets. The intricate molecular mechanisms underlying regulation of platelet aggregation are complex. Glycoprotein layer of the platelet plays a very crucial role in platelet adhesion and aggregation, the various receptor-specific platelet activation signaling pathways converge into common signaling events that stimulate platelet shape change and granule secretion and ultimately induce the “inside-out” signaling process leading to activation of GPIIb/IIIa, then it trigger “outside-in” signaling and acts as a receptor for fibrinogen, von willebrand factor, and fibronectin, resulting in platelet granule secretion, stabilization of platelet adhesion and aggregation [34].

Another interesting finding of this study was that the effect HMGB1 on platelet activation depended the the cGMP signaling pathway. The conclusion is supported by our data that HMGB1decrease cGMP level and the effect of platelet aggregation was abolished by cGMP analogs 8-pCPT-cGMP or cGMP-elevating NO donor SNP which inhibiting platelet activation. At present, regulation of platelets GPIIb-IIIa-integrin activation involving dependent or independent of the NO/cGMP pathway [35]. Most of studtes confirm the concept that the NO/sGC/cGMP/PKG pathway plays excluvely inhibitory roles in platelets [25, 36], however, its effector cGMP also exerts some stimulatory effects on the early phases of activation [37]. The exact mechanisms involved in cGMP-mediated platelet inhibition and the wiring of the cyclic nucleotide signaling network are only partly understood [25]. cGMP production in platelets depends on a single enzyme, the soluble NO-sensitive guanylyl cyclase (sGC or NO-GC), a number of recent studies about cGMP with platelets have demonstrated that stimulation platelet aggregation by blocking the activity of nitric oxide/cGMP signaling or elevating cGMP in the inhibition of platelet aggregation, such as thrombospondin-1 from platelet-granules inhibits cGMP-mediated activation of cGMP-dependent protein kinase induced platelet aggregation [38], activators of cGMP or cAMP inhibition of collagen-induced platelet aggregation [39].

The article "HMGB1: a novel protein that induced platelets active and aggregation via Toll-like receptor-4, NF-κB and cGMP dependent mechanisms" was retracted in 2018. Reasons: errors in the methods; errors in the text; false authorship; unreliable results or conclusions.

In addition, previous disccussion that there is a common regulatory network of inflammation and thrombosis, many studies suggested that HMGB1 play a wide range of biological effects via NF-κB passway, Involving regulation of inflammation, tumor, immune cells’ activation [6, 7, 40], meanwhile, although platelets are anucleated cells, NF-κB is expressed in platelets and that platelet stimulation with agonist triggering IκBα nphosphorylation/degradation, importantly, NF-κB inhibitors are capable of negatively regulating ADP, epinephrine and collagen induced platelet aggregation [41]. Moreover, these also studies suggested that NF-kappa B inhibition of platelet activation dependent the pivotal mechanisms of endothelial nitric oxide synthase/cyclic GMP [42], the mechanism is not very clear about NF-kappa B inhibitors interfere with platelet function.our results indicated NF-kappa B through cGMP signal regulation of HMGB1 induced activation (Fig. 9). The support data is that guanylate cyclase (sGC) inhibitor ODQ can increase IκBα phosphorylation that impaired by BAY 11-7082.

**Fig. 9:** HMGB1 involves in platelets signal pathway

## Conclusion

In conclusion, our data indicated that rHMGB1-induced platelet aggregation and secretion via TLR4 receptors, NF-kappa B, and cGMP depended activation of the GPIIb/IIIa pathway. Together, these experimental data provide evidence for the hypothesis that HMGB1 stimulated platelet activation might play an important role in the haemostasis and thrombotic diseases. This project might provide a new avenue for the treatment of thrombotic diseases via blocking HMGB1 or it’s signal passway in the future.
